# Application of Image Mosaic Technology in Tai Chi Animation Creation

**DOI:** 10.1155/2022/4775189

**Published:** 2022-01-13

**Authors:** Yajun Pang

**Affiliations:** College of Physical Education, Luoyang Institute of Science and Technology, Luoyang, Henan 471023, China

## Abstract

Panorama can reflect the image seen at any angle of view at a certain point of view. How to improve the quality of panorama stitching and use it as a data foundation in the “smart tourism” system has become a research hotspot in recent years. Image stitching means to use the overlapping area between the images to be stitched for registration and fusion to generate a new image with a wider viewing angle. This article takes the production of “Tai Chi” animation as an example to apply image stitching technology to the production of realistic 3D model textures to simplify the production of animation textures. A handheld camera is used to collect images in a certain overlapping area. After cylindrical projection, the Harris algorithm based on scale space is adopted to detect image feature points, the two-way normalized cross-correlation algorithm matches the feature points, and the algorithm to extract the threshold *T* iteratively removes mismatches. The transformation parameter model is quickly estimated through the improved RANSAC algorithm, and the spliced image is projected and transformed. The Szeliski grayscale fusion method directly calculates the grayscale average of the matching points to fuse the image, and finally, the best stitching method is used to eliminate the ghosting at the image mosaic. Data experiments based on Matlab show that the proposed image splicing technology has the advantages of high efficiency and clear spliced images and a more satisfactory panoramic image visual effect can be achieved.

## 1. Introduction

Tai Chi is one of China's precious cultural resources and one of the important cultural industries to promote regional economic development. This article uses animation to promote this cultural product. When using 3D animation production software to design anime character models, in order to save manpower and time, low-precision models can be used. However, in order to achieve exquisite and realistic visual effects for the characters, the real character images are used as the model textures when making the model textures. To make up for the shortcomings of low-precision models. However, the collected real person images need to be spliced into a two-dimensional plane 360° panoramic view according to the requirements of the model UV distribution map, which can be completed by using image splicing technology. Image stitching technology is used in many areas of life. For example, in the field of medical research, with the increasing use of microscopes, pictures under high magnification microscopes are likely to separate the areas that doctors want to observe. The image mosaic technology can be adopted to generate a new mosaic to help doctors solve the problem of not being able to pass one. Other application fields include military field, aerospace field, mechanical design field, and so on. This article will take a group of real person head images as an example to describe the process of using image stitching technology to make 3D model textures [1–5].

Image mosaic technology is an important research topic in the fields of virtual reality, computer graphics, and image processing. In the field of animation, it is used to make animated model textures to save costs and improve the speed and accuracy of making model textures. In the field of TIP (tour into the picture), panoramic images are generated to provide an important basis for generating dynamic three-dimensional images in two-dimensional still images.

Image stitching technology (see Figure 1) is the registration and fusion of several adjacent images or photos with overlapping areas to form a 360-degree or wide-view panoramic image. The image stitching algorithm mainly focuses on the method based on the area correlation and the feature. The method based on the area correlation determines the variance function through the similarity of the images and determines the transformation relationship between the images through the function. This method requires the transformation amplitude between the images to be small, and the method is easy to be affected by care conditions and has a large amount of computer. The feature-based method is to extract the image features and determine the corresponding relationship between the features to find the transformation relationship between the images. This method is relatively stable, fast, and has a wide range of adaptation [6–8].

As one of the important contents of image stitching, image registration is mainly divided into the following.

### 1.1. Registration Based on Image Grayscale

This type of method directly uses image gray information to construct a similarity function for similarity calculation. Commonly used methods are the projection matching method proposed by Fuh CS and the mutual information matching method proposed by P. Viola. The principle of the image registration algorithm based on gray information is simple, but the amount of calculation is large, and because it calculates the gray information of pixels, it is very sensitive to noise and light.

### 1.2. Image Registration Based on Transform Domain

Transform the picture into the frequency domain, and then perform the corresponding transformation processing to realize the image registration, such as the phase correlation matching method based on Fourier transform proposed by Srinivasa and Reddy. The time delay in the time domain corresponds to the phase change in the frequency domain, and the corresponding change in the amplitude is relatively simple, so it is generally used in affine conversion image registration, but it is not suitable for complex graphics conversion forms.

### 1.3. Image Registration Based on Features

Image features include feature points, contour features, regional special diagnosis structure, edge features, and so on. In addition, there are many commercial image stitching software, such as open-source software Hugin, Apple's QuickTime VR system, Microsoft's Digital Image, and so on.

The domestic image splicing technology started later than Europe and America, but it has developed rapidly in recent years. In the field of edge extraction, Wen Ting et al. comprehensively considered the effects of image gradient features, phase features, and noise and used directional energy and the brightness gradient calculated by the histogram difference operator as image features for edge detection; Sun Shuyi et al. used wavelet transform extracts edge features, and then uses manual selection for registration. In terms of feature point extraction, the feature point extraction based on the variational B-spline filter combined with the Harris algorithm proposed by Zhang Yong et al. has significantly improved the time complexity of the algorithm; the tracking grouped Harris proposed by Xu Xianfeng et al. Laplace algorithm feature point extraction has the advantage of reducing feature redundancy; Qiu Guoqing and others improved the Harris algorithm to avoid the *k* value in the corner response function and the selection of the threshold *T* during the detection process [9–12].

Although many scholars at home and abroad have done a lot of research on feature extraction and matching, and have achieved obvious results, the research work on how to improve the speed of feature extraction, improve matching accuracy, reduce redundancy, and enhance robustness is still ongoing. The author thinks that it is difficult to find an algorithm that is suitable for all image stitching, after all, the fields of image stitching are not the same. In the medical field, the emphasis is on the quality of spliced images, because if mismatches, missing matches, and a little ghosting occur, they will have a greater impact on the doctor's judgment; in the aerospace field, the emphasis is on the robustness of spliced images. Great because the objects in the celestial pictures taken are moving and the light is different. In the smart tourism system, due to the high quality of pictures, the focus of algorithm improvement should be to reduce redundancy and reduce the time complexity of the stitching algorithm [13–15].

The main steps of panoramic image production are based on feature points. First, the image with a certain overlapping area is collected, and then the image is preprocessed. According to the stitching method in this article, the image is cylindrically projected, then extract feature points, match feature points, image transformation, and finally generate a panorama through image fusion. Image acquisition is divided into three methods: the camera is placed on a pulley to shoot in parallel, the camera is placed on a tripod to take a fixed rotation, and the camera is held in hand to shoot. This article uses the most common and flexible handheld camera shooting method. This method is widely used and has practical research significance. It is difficult to stitch together images collected by a handheld camera because the camera movement is complicated during the shooting process, and there is a horizontal and vertical offset. There may be a certain exposure difference between adjacent images and a small range of object movement, or even a certain amount in the rotation of the angle and the scaling of the small scale (the scale is the size of the object or feature) [16–23]. The various objects or features of the collected images need to be studied within a specific scale to make sense. A panoramic image is a representation of a discrete image processed into a continuous image. In order not to destroy the visual consistency between various objects in the image and maintain the spatial constraint relationship in the actual scene, the collected discrete images need to be projected onto standard coordinates. According to the form of its projection surface, the panorama can be divided into three types: spherical surface, cube surface, and cylindrical surface. Because the cylindrical projection image is easy to obtain, the image quality is uniform, and the detail is high, it is widely used. This article is an image stitching algorithm that uses a cylindrical surface as the projection surface. After the feature points are extracted, the two-way normalized cross-correlation method is used for feature point matching. The transformation matrix calculation is to calculate the spatial geometric transformation of two images to be spliced according to the feature point matching point set. The transformation matrix model used in this article is an eight-parameter projection transformation model. The model describes the translation, rotation, scaling and regularity of the image stretching also includes irregular stretching, that is, parallel lines cannot remain parallel after transformation. After the image is cylindrically projected, an image matching operation is required, that is, the images of adjacent overlapping areas are spliced and merged. The splicing method based on feature points extracts image feature locations by describing features. This paper adopts a Harris corner detection feature point algorithm with scale spatial information. After the image projection transformation, the image needs to be fused, that is, the coordinates of the reference image and the target image are merged into one coordinate. The directly stitched image often has problems such as grayscale difference and ghosting, which requires the stitched image perform grayscale adjustments and eliminate ghosting operations [24–29].

## 2. Image Stitching

When the “Tai Chi” character image is collected, the postimage stitching and the UV distribution of the character model should be fully considered. In order to obtain a 360° panoramic image of the “Tai Chi” character's head, when the image is collected, the “Tai Chi” character's head is taken as the central axis, and the camera is rotated around the central axis to take a picture. During the shooting process, continuous shooting from multiple angles is required. The lens must be aimed at the head of the person, and there must be a certain degree of overlap between the consecutive images taken. The way of image acquisition is shown in Figure 2.

Image stitching is a complex process, and the main steps of the process can be summarized as: image preprocessing, image projection transformation, image registration, and image fusion.

### 2.1. Image Preprocessing

For cylindrical panoramas, we require the camera to remain still on the horizontal line when capturing images, try to avoid the pitch and tilt of the lens, and perform 360-rotation shooting in the horizontal direction. If conditions permit, place the camera on a fixed tripod, and the effect will be better. The number of pictures taken determines the workload of stitching. The more pictures, the greater the workload. However, if the visual range of the width of each picture is expanded in order to reduce the stitching time, the overlap area between adjacent pictures will be reduced, resulting in inaccurate feature matching and even stitching failure. Weighing the two sides, we generally require that the overlapping area between adjacent pictures be about 50%. Finally, the content to be shot is required to be immobile, that is, there are no moving people or objects; otherwise, it will cause distortion of the stitching graphics or even stitching failure.

Due to the changeable environment, the image will inevitably have noise points. These noise points may cause interference during feature extraction and affect the matching effect and efficiency. Therefore, before the projection transformation, the image is denoised first. Properties such as brightness, color, shape, and grayscale of a set of continuously acquired images vary due to human or natural factors. Therefore, it is necessary to preprocess the problems of low contrast, deformation, geometric distortion, and so on that appear in the image. This will not only improve the display quality of the image but also it can ensure the smooth progress of the subsequent image registration process.

### 2.2. Image Projection

Why do we need to project? Can the overlapping captured images be directly stitched? It can be spliced, but the effect is not ideal. Because the image is the projection of the real scene in two-dimensional coordinates, directly splicing the image cannot meet the human's requirement for visual consistency. Simply put, the pictures taken are horizontal plane imaging, and the pictures we need are cylindrical imaging. Direct stitching will produce distortion.

The biggest feature of the cylindrical panorama is that it has no top and no bottom and can only be used for small-angle pitch operations. This article chooses cylindrical panorama as the research content for the following reasons:

1. The picture collection of the cylindrical panorama is simple
2. The edge distortion of the cylindrical panorama is small, and the pixels are evenly distributed
3. The coordinate transformation of the cylindrical panorama is relatively simple, and there are no edges and fixed points in the cube panorama, so the determination of coordinates and the difficulty of stitching are reduced

Cylindrical panoramas need to project the plane image onto a cylindrical body with the camera focal length *f* as the radius. At the same time, the focal length of the camera needs to be used in the plane and cylindrical coordinate transformation and the calibration of the camera coordinates. The camera focal length *f* is a panorama, which is an important parameter in the generation process. But the focal length parameters of most cameras are not given, especially for pictures taken with mobile phones on the road. Therefore, before the cylindrical projection of the image, we must first estimate the focal length of the shooting camera used.

The images collected according to the method shown in Figure 2 were taken at different angles. In order to maintain the spatial constraint relationship of the actual objects, the collected images need to be projected on a standard coordinate system. Otherwise, if you directly control these images and the splicing is performed, the visual consistency between various objects in the actual scene will be destroyed, and people's visual requirements will not be met. Because the shape of the head profile used in this article is like a cylinder, the projected image has nothing to do with its projected position on the surface of the cylinder. A cylindrical projection model as the standard coordinate space is selected in this article.

As shown in Figure 3, the coordinate system is established with *O* as the origin, I is an original image taken by the camera, where point P (*x*, *y*) is any pixel on the original image *I*, then the pixel point *P* is the coordinates in the camera coordinate system *xyz* can be expressed as

(1) $$\begin{array}{c} \left(x-\frac{W}{2},y-\frac{H}{2},-f\right). \end{array}$$

Here, *W* is the width of the original image *I*, and H is the height of the original image *I*. If the center of the cylinder is used as the origin of the camera's coordinate system, and the camera's pixel focal length *f* is used as the radius of the cylinder, then in a cylindrical panoramic image, the projection point *Q* (*x*′, *y*′) can be expressed as

(2) $$\begin{array}{c} \left\{\begin{array}{c} x^{\prime }=f\;\arctan\left(\frac{x-W/2}{f}\right)+f\;\arctan\left(\frac{W}{2f}\right),\\ y^{\prime }=\frac{f\left(y-H/2\right)}{\sqrt{{\left(x-W/2\right)}^{2}+f^{2}}}+\frac{H}{2}. \end{array}\right. \end{array}$$

Here, *f* is the focal length and satisfies the following formula:

(3) $$\begin{array}{c} f=\frac{W}{2\;\tan\left(hf_{ov}/2\right)}. \end{array}$$

It can be concluded from the formula (2) that the cylindrical projection algorithm can prevent the object from being deformed in the vertical direction.

### 2.3. Image Registration

Image registration uses similarity measures to calculate spatial transformation parameters and transforms two or more pictures of the same scene with a certain degree of similarity from different perspectives and at different times to the same coordinate system to obtain a spliced picture. Image registration has always been the focus of image mosaic technology research, and scholars at home and abroad have also proposed a variety of image registration algorithms. In general, image registration must include the following basic content:

1. Feature space, that is, the collection of features of the image to be matched, such as grayscale features, statistical features (moment invariants, center), edges, corners, etc.: when selecting features, attention should be paid to the number of selected features, too much will increase the amount of matching, and too little will cause matching failures.
2. Selection of similarity measures: it is used to measure the similarity between matching features. It is the most critical step of registration and directly determines the accuracy of matching.
3. Search space, that is, all possible transformation spaces.
4. The best space, which is to find the transformation parameters with the highest similarity in the search space.

Due to the different shooting time of the two images during the stitching process, the gray value of the same scene is not necessarily the same, so stitching will occur at the stitching. The purpose of image fusion is to eliminate seams, make the image naturally excessive, and maintain the good spectral characteristics of the image itself (Figure 4).

The basic principle of image registration is to splice multiple pictures containing the same image area and use a certain matching method for the same image area to determine the splicing position between two adjacent images. Based on the characteristics of a person's head image with rich edge information, texture information, and feature point information, this article adopts the Harris corner detection algorithm based on feature point matching. The corner detection formula is

(4) $$\begin{array}{c} E\left(\Delta x,\Delta y\right)={\sum_{x,y}w\left(x,y\right)\left[I\left(x+\Delta x,y+\Delta y\right)-I\left(x,y\right)\right]}^{2}, \end{array}$$

where *w*(*x*, *y*) is the window function and *I*(*x*+Δ*x*, *y*+Δ*y*) − *I*(*x*, *y*) is the gradient value of the image grayscale. For each small displacement (Δ*x*, Δ*y*), the bilinear approximation can be expressed as

(5) $$\begin{array}{c} E\left(\Delta x,\Delta y\right)≅\left[\Delta x,\Delta y\right]M\left[\begin{array}{c} \Delta x\\ \Delta y \end{array}\right]. \end{array}$$

Here, *M* can be expressed by the following formula:

(6) $$\begin{array}{c} M=\sum_{x,y}w\left(x,y\right)\left[\begin{array}{c} I_{x}^{2}I_{x}I_{y}\\ I_{x}I_{y}I_{y}^{2} \end{array}\right]. \end{array}$$

Let *λ*_1_ and *λ*_2_ be the two eigenvalues of the matrix *M*, representing the curvature of the local autocorrelation function. *E* can be approximated as a local cross-correlation function, describing the shape at this point. When the values of both *λ*_1_ and *λ*_2_ are small, if the window moves in any direction, the change in the value of *E* is small; when one of *λ*_1_ and *λ*_2_ is large, and the other value is small, if the window moves along the edge direction, the change in *E* value is also small, and if the window moves in the direction perpendicular to the edge, the change in *E* value is greater; and when both *λ*_1_ and *λ*_2_ are both large, the moving in any direction will cause the *E* value to increase sharply. The value variation is plotted in Figure 5. According to the above situation, the response function used to calculate the corner point in actual application can be written as

(7) $$\begin{array}{c} R=\det\left(M\right)-{\text{kTrace}}^{2}\left(M\right), \end{array}$$

where

(8) $$\begin{array}{c} \det\left(M\right)=\lambda_{1}\lambda_{2},\text{Trace}\left(M\right)=\lambda_{1}+\lambda_{2}. \end{array}$$

When the determinant of the matrix *M* is large, it indicates that it is an edge or a corner; when the sum of the main diagonals of the matrix *M* in a certain area is large, it indicates that it is an edge. *k* generally takes an empirical value of 0.04.

The Harris corner detection algorithm can extract the feature point information used to register the two images. However, the extracted feature point information cannot be used for matching. It is also necessary to measure the similarity of these feature point information. The performance metric determines the relevant characteristics of all registration tests. First, extract a correlation window of (2*N* + 1) × (2*N* + 1) size in the two images with each feature point as the center, and then use each feature point in the reference image as a reference point, and proceed according to the feature point in the current image. Search sequentially and perform block matching. The search area can be specified during matching, and its range can also be specified according to experimental experience. With this method, the search area of the corresponding feature point can be changed from the entire image to a window of a specified size, which can greatly reduce the calculation Workload. This article uses the normalized cross-correlation (NCC) algorithm to calculate the correlation coefficient between two correlation windows. After the rough matching of feature points above, there are still a small number of false feature pairs. If the least squares method is used to estimate the model parameters directly, it will bring a relatively large registration error. Therefore, this paper uses the RANSAC method to achieve fine matching. This algorithm can effectively exclude outliers in feature matching.

### 2.4. Image Fusion

After the image is spliced, due to the different perspectives, resolutions, etc., of the original image plus the influence of external factors such as lighting, the spliced image will produce blur, noise, or ghost in the overlapped part, and the splicing will occur at the same time. There may also be seams at the borders. Therefore, it is necessary to perform fusion processing on the spliced images. In this article, the multiresolution fusion method is adopted, and the implementation process is as follows:

(1) Create a pyramidal hierarchical structure of the original image to obtain the low-pass layer of each image:
  (9) $$\begin{array}{c} G_{l}\left(x,y\right)=\sum \sum_{m,n=-2}^{2}w\left(m,n\right)G_{l-1}\left(2x+m,2y+n\right). \end{array}$$
Here, *G*_0_ is the original image.
(2) Through the obtained low-pass layer of each image, the bandpass layer of the corresponding image can be decomposed:
  (10) $$\begin{array}{c} L_{l}\left(x,y\right)=G_{l}\left(x,y\right)-4\sum \sum_{m,n=-2}^{2}G_{l}\left(\frac{2x+m}{2},\frac{2y+n}{2}\right). \end{array}$$
(3) Perform the image fusion operation in the bandpass layer of each image separately and use the weighted average method to achieve, then for the current *L*_k_ layer, there are
  (11) $$\begin{array}{c} L_{\text{kout}}\left(x,y\right)=\frac{\sum_{i=0}^{i=N-1}L_{kli}\left(x^{\prime },y^{\prime }\right)w_{i}\left(x^{\prime }\right)w_{i}\left(y^{\prime }\right)}{\sum_{i=0}^{i=N-1}w_{i}\left(x^{\prime }\right)w_{i}\left(y^{\prime }\right)}. \end{array}$$
After this step, the bandpass space corresponding to the output image is obtained.
(4) Combine the obtained bandpass layers to obtain the final stitched image:
  (12) $$\begin{array}{c} G_{\text{out}}=\sum_{k=0}^{N}L_{\text{out}}. \end{array}$$
It can be seen through experiments that the fused image is clear, smooth, and seamless.

## 3. Image Feature Extraction and Matching

The feature of an image is the abstract expression of the pixels or collections of pixels in the image, and it is the most basic attribute that distinguishes the image. It can describe image information with fewer pixels. The feature extraction of the image is chosen because it can avoid the influence of noise, grayscale, and other external factors to a greater extent.

The image features include feature lines, feature faces, feature points, and so on. Special line: the feature line mostly refers to the edge features of the image, including contours and arcs. Usually, edge detection algorithms are used to detect the characteristic curve. The error variation is shown in Figure 6:

  Feature points: feature points are points that reflect the types of features or geographic distribution characteristics of the area. Generally speaking, feature points refer to corner points (currently, there is no clear mathematical definition) or extreme points in the calculated values of other feature extraction functions. The corner points where the boundary direction changes significantly have the greatest probability.
  Feature surface: it refers to the area block that contains the significant information in the image, also called the feature domain. Most of the feature surface extraction is the obvious closed area, and the commonly used extraction method is the segmentation method. The biggest difficulty of image stitching technology based on feature surface lies in the extraction of feature regions.

The matching feature point pairs obtained by the NCC algorithm will have a lot of errors. One is caused by the inaccurate positioning of the feature points. This effect can be reduced when using the least squares method to solve the transformation matrix, and the other is due to interference such as noise. If there are many mismatches, it will have a great influence on the matrix of graph transformation. Therefore, after the NCC matching is completed, the matching pair will be “purified.” Here we introduce the RANSAC algorithm. The image process is shown in Figures 7 and 8.

The RANSAC algorithm is a mathematical model that uses an iterative algorithm to estimate parameters. It is an algorithm with a high fault tolerance rate, combined with the NCC algorithm, it can effectively bring out the external points. The idea of the RANSAC algorithm is to find the transformation model that contains the most interior points through iteration. Taking straight line fitting as an example, we need to find a fitted straight line that contains as many points in the figure as possible. We first select two points, find a straight line, and then take a certain threshold *t*, mark the points with a distance less than *t* from the straight line as interior points, and then find a straight line based on the interior point set obtained this time, and use *t* to judge the same How many points belong to the interior points of the straight line at this time, until a certain sampling makes the number of interior points the largest, and the straight line at this time is the desired one.

For images with a large amount of data, we continue to sample and find the transformation matrix. The *H* matrix determined by every 4 matching points needs to be verified one by one, which is a lot of work. In this article, when using the RANSAC algorithm to purify and calculate the *H* matrix, an improvement is made: 4 + 2 pairs are selected for the initial matching point, and the *H* matrix determined by the 4 feature points is determined by the other 2 pairs of feature points. If they are not all interior points, then just discard it and choose 4 + 2 pairs of matching points.

The images used in the experiment are images collected with a handheld mobile phone under the conditions of fixed-point rotation and translation under outdoor lighting, and the overlap rate of the collected images is about 20%. After the image is collected, the image is first cylindrically projected, the image feature points are extracted using the Harris algorithm with invariant scale space, and the two-way normalized cross-correlation method is used for matching, the feature points are extracted iteratively to remove mismatches, and the projection model is estimated using the RANSAC algorithm, and finally adopt the Szeliski grayscale fusion method. The method of direct gray-level averaging of matching points and the best stitching line completes the mosaic processing of the panorama. Figure 5 is the final stitching effect picture, and the stitching image quality can meet the requirements of TIP background image and animation model texture. The stitched image is shown in Figure 9.

## 4. Conclusion

Image stitching technology is a popular research direction in the field of digital image processing, and it has attracted many scholars to study it in recent decades. Among them, image registration is its key technology. For image registration technology, people generally hope to improve from three aspects, one is the accuracy of feature extraction, the other is the extraction speed, and the third is the accuracy of matching.

In the creation of Tai Chi animation, the pictures that need to be spliced are often portrait pictures, and to achieve a good publicity effect, the quality of the pictures must be relatively high, and there may be more features, which increases the workload of feature matching. Starting from the general direction of saving time, the article sacrifices a small amount of time to reduce the accumulation of feature points that are easy to appear in the classic Harris algorithm, reduces redundancy, reduces the workload for feature matching of the following pictures, and proposes to increase two pairs of matching points. The prejudgment matching matrix greatly reduces the calculation time of the RANSAC algorithm, especially the transformation model calculation for high-quality tourist scenery pictures.

In my country, the National Tourism Administration has included “smart tourism” in the “Twelfth Five-Year Tourism Development Plan.” In a policy-supported environment, the rapid development of Internet of Things technology, cloud computing, modern communication technology, and virtual reality technology related to smart tourism has also provided technical support for it. The popularity of smart phones and tablet computers has also provided them with strong hardware support and user base. Therefore, the development prospects of smart tourism are very good.

The formation of a cylindrical panorama is simpler than that of a spherical panorama, but it cannot be transformed from the top view and the top view, and when roaming, the distortion on both sides is obvious. The matching strategy in this paper is pairwise registration. For multiimage splicing, the matching process is repeated many times, which wastes a lot of time. How to realize the registration and fusion of multiple images together is also a problem that the author considers. The last is the loading of recommended information. Now in the system, the panorama can only be browsed, without any information displayed. Because the cruise ship is very large, the author considers the actual consumption information of previous passengers and the click-through rate of each panorama as the criterion and adds recommended stars to the panorama to make the purpose of tourist's cruise clearer.

## Figures and Tables

**Figure 1:** Image stitching technology.

**Figure 2:** The way of image acquisition.

**Figure 3:** Coordinate system.

**Figure 4:** Value with different data.

**Figure 5:** Value variation.

**Figure 6:** Error variation.

**Figure 7:** Image process.

**Figure 8:** Process data.

**Figure 9:** The stitched image.

## Data Availability

The data set can be accessed upon request to the corresponding author.
